# Intrauterine Growth Retardation Affects Intestinal Health of Suckling Piglets via Altering Intestinal Antioxidant Capacity, Glucose Uptake, Tight Junction, and Immune Responses

**DOI:** 10.1155/2022/2644205

**Published:** 2022-03-19

**Authors:** Xiaopeng Tang, Kangning Xiong

**Affiliations:** ^1^School of Karst Science, Guizhou Normal University, No. 116 North Baoshan Road, Yunyan District, Guiyang 550001, China; ^2^State Engineering Technology Institute for Karst Desertification Control, No. 116 North Baoshan Road, Yunyan District, Guiyang 550001, China

## Abstract

The aim of the present study was to investigate the effects of intrauterine growth retardation (IUGR) on the intestinal morphology, intestinal epithelial cell apoptosis, intestinal antioxidant capacity, intestinal glucose absorption capacity, and intestinal barrier function of piglets during the suckling period. A total of eight normal-birth-weight (NBW) piglets and eight IUGR newborn piglets (Duroc × Landrace × Yorkshire) were selected from eight litters, one NBW and one IUGR newborn piglet per litter. In each litter, piglets with birth weight of 1.54 ± 0.04 kg (within one SD of the mean birth weight) were selected as NBW piglets and piglets with birth weight of 0.82 ± 0.03 kg (two SD below the mean birth weight) were selected as IUGR piglets. At 21 days of age, all piglets were killed by exsanguinations for sampling. The results showed the body weight (BW) of IUGR piglets on day 0, day 7, day 14, and day 21, and the body weight gain (BWG) of IUGR piglets was significantly lower than that of NBW piglets. IUGR piglets exhibited impaired intestinal morphology, raised enterocyte apoptosis, and increased oxidative damage. It showed that IUGR leads to a lower antioxidant capacity and glucose absorption in the jejunum. In accordance, IUGR caused the intestinal barrier dysfunction by impairing tight junctions and increasing intestinal inflammatory injury. Collectively, these results add to our understanding that IUGR affects intestinal health of suckling piglets via altering intestinal antioxidant capacity, glucose uptake, tight junction, and immune responses, and the slow growth of piglets with IUGR may be associated with intestinal injury.

## 1. Introduction

Intrauterine growth retardation (IUGR) is usually defined as a failure of normal growth and development of a mammalian embryo/fetus or its organs during pregnancy, which has become a difficult problem in human medicine and animal husbandry [1, 2]. Animals with IUGR are characterized by feeding intolerance and gut dysfunction, which negatively influences neonatal survival, postnatal growth, feed utilization, and normal function of tissues or organs [3, 4]. As a kind of common domestic mammal animal with multiple pregnancies, pigs have a high incidence of IUGR (about 15%-20%), which would cause considerable economic losses in large-scale pig production farms [1, 5]. Therefore, a good understanding of the characteristics of intestinal injury in IUGR piglets is of prime importance to improve the growth performance and health status of IUGR animals. Meanwhile, due to the high similarities between pigs and humans in anatomy, physiology, and nutrient metabolism, IUGR pigs can be used as an ideal animal model to study human diseases [6, 7].

The suckling period is an important stage for the continuous improvement of intestinal digestive function, the gradual maturity of the immune system, and the early colonization of intestinal microorganisms, which has a profound impact on the growth and development of animals [8]. Previous studies had confirmed that IUGR could cause impaired development of the gastrointestinal tract of piglets, which is manifested by decreased intestinal length and weight [9], decreased villus height (VH) and increased crypt depth (CD) [10], increased apoptosis of intestinal epithelial cells [11], and increased oxidative damage [12]. The delay and alteration of gut development of IUGR piglets are likely to play a major role in poor adaptability, slow growth, and high morbidity and mortality after birth [13].

Normally, oxidative stress and damage are due to high concentrations of reactive oxygen species (ROS), and the negative effects can be balanced by antioxidant defense mechanisms, including nonenzymatic antioxidant systems (such as ascorbic acid, vitamin E, and glutathione) and enzymatic antioxidant systems, such as superoxide dismutase (SOD), catalase (CAT), and glutathione peroxidase (GSH-Px) [14]. Previous studies revealed that IUGR could impair intestinal morphology and cause serious oxidative damage [12, 15], which may result in a poor intestinal absorption of nutrients, such as glucose. Intestinal health of piglets at the end of lactation is critical to postweaning adaptation. However, studies that describe the intestinal health of IUGR neonatal piglets at the end of lactation are currently very limited. Therefore, in the present study, we chose IUGR piglets as animal model to investigate the effects of IUGR on intestinal health of piglets from the aspects of intestinal antioxidant capacity, glucose absorption, and intestinal barrier function.

## 2. Materials and Methods

### 2.1. Animals and Experimental Design

The experimental procedures involving animals were approved by the animal welfare committee of the Guizhou Normal University (Guiyang, China). The sows with similar birth order (third or fourth) were fed with the same gestating diet. On the day of delivery, the body weight of each newborn piglet was recorded. A total of eight normal-birth-weight (NBW) and eight IUGR newborn piglets (Duroc × Landrace × Yorkshire) were selected from eight litters (4 males and 4 females), one NBW and one IUGR newborn piglet per litter. In each litter, piglets with birth weight of 1.54 ± 0.04 kg (within one SD of the mean birth weight) were selected as NBW piglets and piglets with birth weight of 0.82 ± 0.03 kg (two SD below the mean birth weight) were selected as IUGR piglets. During suckling, selected NBW and IUGR piglets were suckled by their mother sows to 21 days of age. The body weight (BW) of the piglets was recorded at days of 0, 7, 14, and 21 to observe the average body weight gain (BWG) of the piglets during suckling.

### 2.2. Sample Collection

At 21 days of age, blood was obtained by jugular venipuncture and then centrifuged at 3000 × *g* for 15 min at 4°C to obtain serum samples (*n* = 8). All pigs were exsanguinated after being anaesthetized with an injection of sodium pentobarbital (50 mg kg^−1^ BW). One piece of jejunum segment was fixed in 10% neutral buffered formalin for examination of intestinal morphology (*n* = 8). Jejunum mucosa samples were collected from the middle jejunum and then immediately frozen in liquid nitrogen and stored at −80°C for subsequent analysis (*n* = 8), among which four jejunum mucosa samples (2 males and 2 females) were used for real-time PCR analysis (*n* = 4). The jejunal mucosa was homogenized in ice-cold PBS and then centrifuged at 10000 × *g* for 10 min at 4°C. The supernatant was collected, and the protein concentration was determined using the bicinchoninic acid (BCA) protein assay reagent according to the instructions of the manufacturer (Nanjing Jiancheng Bioengineering Institute, Nanjing, China).

### 2.3. Intestinal Histomorphology

Paraffin sections (approximately 5 mm) of jejunum samples were stained with hematoxylin and eosin, and VH and CD were measured using a light microscope with a computer-assisted morphometric system (BioScan Optimetric, BioScan Inc., Edmonds, WA, USA) according to a previous study [16].

### 2.4. Flow Cytometry

The apoptosis of jejunum mucosa cells was measured by flow cytometry according to previous study [14]. Gently scrape the jejunum mucosa with a clean glass slide, place it in ice-cold phosphate-buffered saline (PBS, Solarbio, Beijing, China), wash with PBS twice, and prepare into 1 × 10^6^ cell/mL single cell suspension. Collected cells were incubated with 10 *μ*M Annexin V-FITC and propidium iodide (PI) (Annexin V-FITC/PI kits) for 15 min at room temperature in the dark. Apoptotic cells were identified using a BD FACSCalibur flow cytometer (BD Biosciences, San Diego, CA, USA). The data were analyzed using the CELLQuest software.

### 2.5. Serum and Jejunal Antioxidant Capacity of Suckling Piglets

Serum and jejunum antioxidant indices, including total SOD (SOD Assay Kit, no. A001-3-2), GSH-Px (GSH-Px Activity Testing Kit, no. A005-1-2), total antioxidant capacity (T-AOC Activity Testing Kit, no. A015-2-1), and malonaldehyde (MDA Concentration Testing Kit, no. A003-1-2), were measured according to the instructions of the manufacturer (Nanjing Jiancheng Bioengineering Institute, Nanjing, China).

### 2.6. ELISA Analysis of Immunoglobulins and Cytokines

The secreted immunoglobulin (sIgA) and cytokines including interleukin 1*β* (IL-1*β*), IL-6, and tumor necrosis factor (TNF-*α*) in jejunum mucosa were measured using enzyme-linked immunosorbent assay (ELISA) kits (Cusabio Biotech Co., Wuhan, China) according to the manufacturer's instructions.

### 2.7. AKP and Na^+^/K^+^-ATPase Activity in Jejunum Mucosa

Jejunum mucosa alkaline phosphatase (AKP) was measured using an alkaline phosphatase assay kit (no. A059-2-2), and sodium/potassium-transporting adenosine triphosphatase (Na^+^/K^+^-ATPase) activity was measured using the Na^+^/K^+^-ATPase assay kit (no. A070-2-2) according to the instructions of the manufacturer (Nanjing Jiancheng Bioengineering Institute, Nanjing, China).

### 2.8. Real-Time PCR Analysis of Gene Expression

The mRNA expression of *SGLT1*, *GLUT2*, *AMPK-α1*, *ZO-1*, *Claudin-1*, and *Occludin* was analyzed by real-time quantitative RT-PCR as described previously [17]. The primers of genes (Sangon Biotech, Shanghai, China) are shown in Table 1. *β*-Actin was used as a housekeeping gene to normalize the target gene expression. The formula 2-^(*ΔΔ*Ct)^, where ΔΔCt = (Ct_Target_–Ct_*β*−actin_) treatment − (Ct_Target_–Ct_*β*−actin_) control, was used to calculated the relative gene expression [16].

### 2.9. Statistical Analysis

The experimental data were performed using Shapiro-Wilk of IBM SPSS statistics 21.0 (SPSS, Inc., Chicago, IL, USA) to test data of normal distribution, and *P* > 0.05 was considered the data are normally distributed. Then, the statistical analysis between the two groups was performed by Student's *t*-test of IBM SPSS statistics 21.0. The results were presented as the mean ± standard error of the mean (SEM). The results of all data analyses were input into GraphPad Prism 7.0 (GraphPad Software, Inc., San Diego, CA) software for graphical display. Mean values were considered to be significantly different when *P* < 0.05.

## 3. Results

### 3.1. Growth Performance

The effects of IUGR on weight gain of piglets during the suckling period are listed in Figure 1. It showed that the BW of IUGR piglets on day 0, day 7, day 14, and day 21 were significantly lower (*P* < 0.05) than those of NBW piglets (Figure 1(a)); the BWG of IUGR piglets were significantly lower (*P* < 0.05) than those of NBW piglets (Figure 1(b)). It means that IUGR had a significantly negative effect on weight gain of piglets during the suckling period.

### 3.2. Intestinal Histomorphology

The effects of IUGR on intestinal morphology are presented in Figure 2. In comparison with NBW piglets, the IUGR piglets exhibited a decrease (*P* < 0.05) of VH and the ratio of villous height to crypt depth (VCR). It also showed that there was a tendency (*P* = 0.083) to increase the jejunum CD of IUGR piglets compared to NBW piglets.

### 3.3. Intestinal Damage Caused by IUGR

To determine the effects of IUGR on intestinal damage, the apoptosis of mucosa cells and oxidative damage in the jejunum was measured. The flow cytometry results showed that the apoptosis of jejunum mucosa cells was higher (*P* < 0.05) in IUGR piglets than in NBW piglets (Figures 3(a) and 3(b)). IUGR could cause a serious intestinal oxidative injury, which is indicated by a higher (*P* < 0.05) MDA level in serum (Figure 3(c)) and jejunum intestine (Figure 3(d)).

### 3.4. Antioxidant Activities

The effects of IUGR on serum and intestinal antioxidant property are presented in Figure 4. Compared with the NBW piglets, the IUGR piglets had a lower (*P* < 0.05) T-AOC level (Figure 4(a)), GSH-Px activity (Figure 4(b)), and SOD activity (Figure 4(c)) in serum and a lower (*P* < 0.05) T-AOC level (Figure 4(e)), GSH-Px activity (Figure 4(f)), SOD activity (Figure 4(g)), and CAT activity (Figure 4(h)) in the jejunum.

### 3.5. Glucose Absorption Capacity

To determine the effects of IUGR on glucose absorption capacity, AKP and Na^+^/K^+^-ATPase activity and *SGLT1*, *GLUT2*, and *AMPK-α1* gene expression were measured. The results showed that the AKP activity (Figure 5(a)), Na^+^/K^+^-ATPase activity (Figure 5(b)), and *SGLT1* (Figure 5(c)) and *AMPK-α1* (Figure 5(e)) mRNA expression in jejunum mucosa decreased significantly (*P* < 0.05) when piglets suffered from IUGR, while there was no difference in the expression of *GLUT2* (Figure 5(d)) between the NBW piglets and IUGR piglets.

### 3.6. Tight Junctions

The effects of EGF on gene expression of tight junctions (*ZO-1*, *Claudin-1*, and *Occludin*) in jejunum mucosa of piglets are presented in Figure 6. The results showed that, compared with the NBW piglets, the IUGR piglets had a lower (*P* < 0.05) gene expression of *ZO-1* (Figure 6(a)) and *Occludin* (Figure 6(c)) in jejunum mucosa, as well as a tendency (*P* = 0.056) to decrease the gene expression of *Claudin-1* (Figure 6(b)).

### 3.7. Immune Response

To determine the immune function in the jejunum mucosa of NBW and IUGR piglets, sIgA and proinflammatory cytokines (IL-1*β*, IL-6, and TNF-*α*) were measured using enzyme-linked immunosorbent assay (ELISA) methods. The results showed that the sIgA level (Figure 7(a)) in jejunum mucosa decreased significantly (*P* < 0.05), while IL-1*β* (Figure 7(b)) and TNF-*α* (Figure 7(c)) increased significantly (*P* < 0.05) when piglets suffered from IUGR. There was no difference in IL-6 (*P* = 0.4218) between the NBW group and the IUGR group (Figure 7(d)).

## 4. Discussion

The birth weight of newborn piglets is an important index in large-scale pig farm, largely because it is positively correlated with survival rate and weaning weight of pigs [18, 19]. IUGR impairs the growth and development of the fetus and is ultimately characterized by a low birth weight. In the present study, IUGR significantly reduced BW and BWG in the whole suckling period (day 0 to day 21), which were consistent with the previous studies that IUGR piglets showed a lower birth weight [4] and weaning weight [20], a slow growth before [20, 21] and after weaning [4, 5, 22] compared to NBW piglets. Previous studies as well as the present study all confirmed that IUGR have an adverse effect on growth performance of piglets.

The intestinal tract is not only an important organ for nutrients digestion, absorption, and metabolism but also an important barrier for animals to prevent the toxins, allergens, and pathogens from the external environment into the circulation system [23–25]. The integrity of morphology and function of the intestine is critical to intestinal health and the utilization of nutrients. So, the slow growth of piglets with IUGR may be associated with intestinal injury. To verify the above hypothesis, we chose 21-day-old IUGR piglets as animal model to investigate the effects of IUGR on intestinal morphology, intestinal epithelial cell apoptosis, intestinal oxidative damage and antioxidant capacity, intestinal glucose absorption capacity, intestinal tight junctions, and immune response.

Substantial evidence has indicated that IUGR is associated with impaired intestinal development [9, 26, 27]. Intestinal morphology which is often evaluated by VH, CD, and VCR can reflect the intestinal development and function [28]. In the present study, the IUGR piglets exhibited a decrease of VH and VCR and an increase tendency of CD in the jejunum. These results are consistent with previous studies who also reported IUGR damage to the intestinal morphology of piglets [13, 26, 27, 29]. The integrity of intestinal morphology is regulated by both cell proliferation and apoptosis [14, 30]. The balance between intestinal epithelial cellular proliferation and apoptosis is necessary to maintain the intestinal barrier function [14]. In the present study, piglets with IUGR had a higher apoptosis rate in jejunum epithelial cells than NBW piglets, which is similar to previous studies that IUGR increased cell apoptosis in the small intestine of neonatal piglets [31], weaned piglets [27], and rats [32].

Oxidative stress is widely recognized as a state of imbalance of oxidation and antioxidation, which has been widely implicated in intestinal epithelium apoptosis [14, 33, 34]. MDA is the primary product of lipid peroxidation and usually considered as one of the markers of oxidative stress [35]. The increased level of MDA in serum and jejunum in the present study indicated that IUGR caused intestinal oxidative damage, which is similar to the previous study who also reported that IUGR can increase the content of MDA in jejunum mucosa of pigs [36]. SOD, GSH-Px, and CAT activities antioxidant enzymes are important indicators of antioxidant function [37, 38]. Previous studies have demonstrated that IUGR increased oxidative stress by decreasing the activities of antioxidant enzymes, such as GSH-Px, SOD, and CAT [4, 12, 15, 26, 36]. We also found that IUGR significantly decreased the activities of antioxidant enzymes of GSH-Px, SOD, and CAT. Numerous studies have demonstrated that oxidative stress is associated with many pathological conditions, including intestinal barrier dysfunction and various digestive tract diseases [14, 39–41]. Therefore, alleviating the negative effects of oxidative stress damage is crucial for the development of IUGR newborn piglets.

It is commonly accepted that glucose is the main carbon and energy source of animals and the small intestine is an important site for glucose absorption [42]. SGLT1, GLUT2, AMPK-*α*1, AKP, and Na^+^/K^+^-ATPase play important roles in glucose absorption in the small intestine. SGLT1, a high-affinity and low-transport-capacity glucose transporter, is the primary carrier protein responsible for the absorption of glucose from the lumen of the intestine across the brush border membrane of intestinal epithelial cells, which is dependent on Na^+^/K^+^-ATPase for energy supply [42–45]. GLU2, a low-affinity and high-transport-capacity glucose transporter, can mediate the intracellular glucose transporter to portal vein [42, 43, 45]. AKP is a key enzyme in intestinal digestion and absorption, which can accelerate the uptake and transfer of nutrients and provide energy for the body indirectly [46]. AMPK is a key molecule in the regulation of biological energy metabolism and has been demonstrated to play important roles in the regulation of cellular glucose uptake through the stimulation of SGLT1 and GLUT2 [47–49]. In the present study, piglets with IUGR had a lower AKP and Na^+^/K^+^-ATPase activity and a lower *SGLT1* and *AMPK-α1* mRNA expression in jejunum mucosa while there was no difference in the expression of *GLUT2* compared to NBW piglets. These results indicated that IUGR negatively affects the intestinal glucose absorption capacity, through inhibiting the expression of *AMPK-α*, thereby reducing express SGLT1 transporters but not GLU2 transporters. Previous studies revealed that the continuous impairment of intestinal development of piglets with IUGR would result in a poor intestinal nutrient absorption capacity by inhibiting the expression of proteins involved in key biological processes such as nutrient absorption, digestion, and transport and protein synthesis in the small intestine of newborn and preweaning piglets [2, 5, 50, 51], which are similar to the present study.

Tight junctions including zonula occludens (ZO-1, ZO-2, and ZO-3), Claudins, Occludin, and junctional adhesion molecule (JAM) are important components of the intestinal mechanical barrier, which is critical in protecting the intestinal barrier function, reducing the intestinal permeability, and preventing bacteria endotoxin and toxic macromolecules' entry into the body [23, 36]. In the present study, the IUGR piglets had a lower gene expression of *ZO-1* and *Occludin* in jejunum mucosa than NBW piglets. Similar result also found that the *Occludin* mRNA expression in the IUGR growing pigs was lower than that in NBW pigs [36]. These results indicated that IUGR damaged the intestinal barrier function by decreasing the transcription of tight junction genes.

In addition, the immune and inflammatory response is closely associated with intestinal barrier function [52, 53]. sIgA, an immunoglobulin secreted by plasma cells of the intestinal mucosa, is a major effector of the intestinal mucosal immunity, which acts as the first defense line to prevent the colonization of pathogens in the intestinal mucosa and plays an important role in local anti-infection of the body [24, 54]. Our results from the present study showed that the sIgA content in jejunum mucosa significantly decreased when piglets suffered from IUGR, which indicated that IUGR damages the intestinal immune function. It was reported that excessive intestinal epithelial cell apoptosis and uncontrolled oxidative stress in the intestine could result in intestinal dysfunction, thereby leading to the inflammatory response and release of proinflammatory cytokines, such as IL-1*β*, IL-6, and TNF-*α* [26, 27, 55]. The results of the present study suggested that IUGR enhanced the concentrations of proinflammatory cytokines (IL-1*β* and TNF-*α*) in the jejunum. Similar to our study, Niu et al. [27] reported that weaned piglets with IUGR had a higher IL-1*β*, IL-6, and TNF-*α* concentrations than NBW weaned piglets; Yan et al. [36] showed that pigs in the IUGR group had a higher mRNA expression of *TNF-α*, *IL-6*, and *IFN-γ* than NBW pigs; Huang et al. [56] demonstrated that piglets with IUGR have increased TNF-*α* and IL-6 level at birth, and Wang et al. [57] also showed that the mRNA expression of *TNF-α* in IUGR piglets was higher than that in NBW piglets. All these studies as well as our study could indicate that IUGR caused swine intestinal inflammatory injury.

## 5. Conclusions

In conclusion, the present results showed that IUGR had a significantly negative effect on growth performance of piglets during the suckling period. Meanwhile, IUGR could cause intestinal injury in the jejunum of suckling piglets, which is indicated by injured intestinal morphology and tight junctions, increased apoptosis of enterocytes, increased oxidative damage, decreased glucose absorption capacity, reduced jejunum immunity, and increased intestinal inflammatory injury. Collectively, these results add to our understanding that the slow growth of piglets with IUGR may be associated with intestinal injury.

## Figures and Tables

**Figure 1:** Effects of intrauterine growth retardation on growth performance of suckling piglets (0 to 21 days). (a) Body weight of piglets at days 0, 7, 14, and 21. (b) Average body weight gain of piglets. Values are expressed as means ± SEM, *n* = 8. NBW: normal-birth-weight piglets; IUGR: intrauterine growth retardation piglets. ^∗^*P* < 0.05 compared with the NBW group.

**Figure 2:** Effects of intrauterine growth retardation on the jejunum morphology of suckling piglets: (a) intestinal morphology of the jejunum, (b) villus height of the jejunum, (c) crypt depth of the jejunum, and (d) the ratio of villus height to crypt depth. Values are expressed as means ± SEM, *n* = 8. NBW: normal-birth-weight piglets; IUGR: intrauterine growth retardation piglets. ^∗^*P* < 0.05 compared with the NBW group.

**Figure 3:** Effects of intrauterine growth retardation on intestinal damage of suckling piglets. (a) Representative charts of flow cytometry analyses of apoptosis. (b) Apoptosis rate. (c) MDA content in serum. (d) MDA content in the jejunum. Values are expressed as means ± SEM, *n* = 8. NBW: normal-birth-weight piglets; IUGR: intrauterine growth retardation piglets. ^∗^*P* < 0.05 compared with the NBW group.

**Figure 4:** Effects of intrauterine growth retardation on serum and intestinal antioxidation capacity of suckling piglets. (a) T-AOC level in serum. (b) GSH-Px level in serum. (c) SOD level in serum. (d) CAT level in serum. (e) T-AOC level in the jejunum. (f) GSH-Px level in the jejunum. (g) SOD level in the jejunum. (h) CAT level in the jejunum. Values are expressed as means ± SEM, *n* = 8. NBW: normal-birth-weight piglets; IUGR: intrauterine growth retardation piglets. ^∗^*P* < 0.05 compared with the NBW group.

**Figure 5:** Effects of intrauterine growth retardation on intestinal glucose absorption capacity of suckling piglets. (a) Alkaline phosphatase (AKP) activity. (b) Sodium/potassium-transporting adenosine triphosphatase (Na^+^/K^+^-ATPase) (*n* = 8). (c) *SGLT1* mRNA relative expression. (d) *GLUT2* relative expression. (e) *AMPK-α1* relative expression (*n* = 4). Values are expressed as means ± SEM. NBW: normal-birth-weight piglets; IUGR: intrauterine growth retardation piglets. ^∗^*P* < 0.05 compared with the NBW group.

**Figure 6:** Effects of intrauterine growth retardation on intestinal tight junction's gene expression of suckling piglets. (a) *ZO-1* mRNA relative expression. (b) *Claudin* relative expression. (c) *Occludin* relative expression. Values are expressed as means ± SEM, *n* = 4. NBW: normal-birth-weight piglets; IUGR: intrauterine growth retardation piglets. ^∗^*P* < 0.05 compared with the NBW group.

**Figure 7:** Effects of intrauterine growth retardation on intestinal immune function of suckling piglets: (a) sIgA level, (b) IL-1*β* level, (c) TNF-*α* level, and (d) IL-6 level. Values are expressed as means ± SEM, *n* = 8. NBW: normal-birth-weight piglets; IUGR: intrauterine growth retardation piglets. ^∗^*P* < 0.05 compared with the NBW group.

**Table 1:** Primers used for quantitative reverse transcription PCR.

Gene	Primers sequence	Product length
*β-Actin*	F: 5′-CATCCTGCGTCTGGACCTGG-3′ R: 5′-TAATGTCACGCACGATTTCC-3′	116 bp
*SGLT1*	F: 5′-ATATGCCCTTATATTCCCCTT-3′ R: 5′-AAATCGTGTTGATAGCGCCAA-3′	138 bp
*GLUT2*	F: 5′-CAGCCTATTCTAGTAGCACTG-3′ R: 5′-AAATCGTGTTGATAGCGCCAA-3′	151 bp
*AMPK-α1*	F: 5′-GGTGAAAATCGGCCACTACA-3′ R: 5′-TTGCCAACCTTCACTTTGCC-3′	72 bp
*ZO-1*	F: 5′-TGCTGGCACTGACCAACGTA-3′ R: 5′-CACTGGGCATAATTCAGACGA-3′	129 bp
*Claudin-1*	F: 5′-TCCTGCTGGGACTAATAGCCAT-3′ R: 5′-CAATGACAGCCATCCGCATC-3′	102 bp
*Occludin*	F: 5′-CATTGCCATTGTACTAGGGTT-3′ R: 5′-GCTGCTCGTCATAAATACGTT-3′	140 bp

## Data Availability

The data used to support the findings of this study are included within the article.
